The article "Cost-Effectiveness Analysis of Biopharmaceuticals for Treating Rheumatoid Arthritis: Infliximab, Adalimumab, and Etanercept" was published in 2021. Journal: Biomed Res Int.

# Cost-Effectiveness Analysis of Biopharmaceuticals for Treating Rheumatoid Arthritis: Infliximab, Adalimumab, and Etanercept

**DOI:** 10.1155/2021/4450162

**Published:** 2021-11-28

**Authors:** Ahmad Gholami, Jassem Azizpoor, Elham Aflaki, Mehdi Rezaee, Khosro Keshavarz

**Affiliations:** ^1^Pharmaceutical Sciences Research Center, Shiraz University of Medical Sciences, Shiraz, Iran; ^2^Biotechnology Research Center, Shiraz University of Medical Sciences, Shiraz, Iran; ^3^Department of Pharmaceutical Biotechnology, School of Pharmacy, Shiraz University of Medical Sciences, Shiraz, Iran; ^4^Department of Rheumatology, School of Medicine, Shiraz University of Medical Sciences, Shiraz, Iran; ^5^Department of Health Management, Policy and Economics, Faculty of Management and Medical Information Sciences, Kerman University of Medical Sciences, Kerman, Iran; ^6^Health Human Resources Research Center, Department of Health Economics; School of Health Management and Information Sciences, Shiraz University of Medical Sciences, Shiraz, Iran; ^7^Emergency Medicine Research Center, Shiraz University of Medical Sciences, Shiraz, Iran

## Abstract

**Introduction:**

Rheumatoid arthritis (RA) is a chronic progressive inflammatory disease that causes joint destruction. The condition imposes a significant economic burden on patients and societies. The present study is aimed at evaluating the cost-effectiveness of Infliximab, Adalimumab, and Etanercept in treating rheumatoid arthritis in Iran.

**Methods:**

This is a cost-effectiveness study of economic evaluation in which the Markov model was used. The study was carried out on 154 patients with rheumatoid arthritis in Fars province taking Infliximab, Adalimumab, and Etanercept. The patients were selected through sampling. In this study, the cost data were collected from a community perspective, and the outcomes were the mean reductions in DAS-28 and QALY. The cost data collection form and the EQ-5D questionnaire were also used to collect the required data. The results were presented in the form of an incremental cost-effectiveness ratio, and the sensitivity analysis was used to measure the robustness of the study results. The TreeAge Pro and Excel softwares were used to analyze the collected data.

**Results:**

The results showed that the mean costs and the QALY rates in the Infliximab, Adalimumab, and Etanercept arms were $ 79,518.33 and 12.34, $ 91,695.59 and 13.25, and $ 87,440.92 and 11.79, respectively. The one-way sensitivity analysis confirmed the robustness of the results. In addition, the results of the probabilistic sensitivity analysis (PSA) indicated that on the cost-effectiveness acceptability curve, Infliximab was in the acceptance area and below the threshold in 77% of simulations. The scatter plot was in the mentioned area in 81% and 91% of simulations compared with Adalimumab and Etanercept, respectively, implying lower costs and higher effectiveness than the other two alternatives. Therefore, the strategy was more cost-effective.

**Conclusion:**

According to the results of this study, Infliximab was more cost-effective than the other two medications. Therefore, it is recommended that physicians use this medication as the priority in treating rheumatoid arthritis. It is also suggested that health policymakers consider the present study results in preparing treatment guidelines for RA.

## 1. Introduction

Rheumatoid arthritis (RA) is a progressive inflammatory disease characterized by inflammation of the synovial membrane and may eventually lead to joint destruction [1, 2]. Due to its long-term chronic and safety course, it is immediately required to treat with immunomodulatory medications [3]. This debilitating condition is supposed to affect 0.3-1.2% of the world's population [4]. Uncontrolled RA leads to progressive joint destruction and performance reduction [5]. These conditions impose a significant underlying economic burden, reduce the quality of life (QOL), and lead to productivity loss [6]. Disease-modifying antirheumatic medications (DMARDs) such as Methotrexate, Sulfasalazine, and Hydroxychloroquine may delay the disease progression [7]. However, many patients do not achieve an appropriate response, and some do not maintain a reaction due to ineffectiveness or toxicity [8].

Nowadays, physicians are trying to achieve less disease activity or, preferably, recovery, rather than simply slowing the progression of the disease and controlling the symptoms [9]. Biopharmaceuticals are drugs that are obtained from biological sources by biotechnological methods [10–12]. The more important these drugs become in medicine, the more attention is paid to concerns such as biosimilars, cost-effectiveness, and price control. The therapeutic value of biopharmaceuticals for the healthcare system is not yet well understood, and this only happens when policymakers understand the effects of these biological products on the economic system of healthcare facilities [13, 14]. The discovery of biopharmaceuticals leads to a dramatic change in the therapeutic approach to RA and results in better QOL [15]. However, success requires the purchase of these medications at high prices [4, 5], which may ultimately increase the financial burden that RA imposes on the community. Such a scenario represents the need for pharmacoeconomics evaluations to inform policymakers and decision-makers about the cost-effectiveness of biological DMARDs [5, 16].

TNF inhibitors are a class of biopharmaceuticals applicable for treating Crohn's disease, ulcerative colitis, rheumatoid arthritis, ankylosing spondylitis, psoriatic arthritis, plaque psoriasis, and/or juvenile idiopathic arthritis. According to the FDA, this category of medicines includes Infliximab, Etanercept, Adalimumab, Certolizumab pegol, and Golimumab. Although the side effects of these medicines are not yet fully understood, several side effects are still under investigation. Some of these well-known adverse effects are bacterial, fungal, viral, or atypical infections, the risk of malignancies, especially lymphomas, congestive heart failure NYHA Class III or IV, drug-induced lupus demyelinating disorders, including optic neuritis, multiple sclerosis, and local injection site reaction/erythema. Infliximab is a chimeric monoclonal antibody composed of fixed human and variable mouse regions [17]. This medication can only be used intravenously and should be used in combination with Methotrexate if possible. The starting dose of the medicine is 3 mg per kg of body weight and can be increased up to 10 mg/kg with an interval of 4-8 weeks. In mid-2001, the FDA/EMA approved Infliximab combined with Methotrexate to treat RA [18].

Infliximab inhibits TNF-*α* binding to its target receptors and prevents the production of other proinflammatory cytokines, including interleukin and GCSF [19]. Common side effects of infliximab therapy include acute injection reactions, infections, and delayed hypersensitivity reactions. The medication is contraindicated in people with moderate to severe heart failure and tuberculosis or other severe or opportunistic infections [20]. Adalimumab is a recombinant human IgG1 monoclonal antibody with no mouse ingredient produced by phage display technology. The FDA/EMA approved it in 2002 to treat moderate to severe RA to be used alone or in combination with other DMARDs. Adalimumab is injected subcutaneously every two weeks [21]. The common side effects of the medication include injection reactions and site infection. Adalimumab is contraindicated in people with moderate to severe heart failure and active TB or people with other severe or opportunistic infections. Before starting the treatment, physicians should examine the patients for active and inactive (latent) tuberculosis infection [20]. Etanercept is also a recombinant human TNF receptor fusion protein that attenuates the effects of endogenous TNF by competitively inhibiting its interaction with cell surface receptors. Etanercept has been proved to be effective in patients with rheumatoid arthritis and is injected subcutaneously at 25 or 50 mg once or twice a week [22].

Considering different medical costs, medication of various financial and economic consequences of these biopharmaceuticals is not clear on the health system, and there is limited knowledge about their cost-effectiveness. Since the researchers could not find any studies that have compared these medications' cost-effectiveness, the present study was conducted to determine and compare the cost-effectiveness of Infliximab, Adalimumab, and Etanercept for patients with RA.

## 2. Materials and Methods

This is a cross-sectional study for the economic evaluation of cost-effectiveness in patients with RA in Fars province in 2019. The study population included all the patients with RA referred to the rheumatology department of Hafez Hospital and the rheumatologists' offices in 2019 and who were treated with one of the following three medications: Adalimumab, Infliximab, and Etanercept. The sample sizes of the patients treated with Adalimumab, Infliximab, and Etanercept based on previous studies, 80% power, and 5% error using the NCSS statistical software were 48, 53, and 53, respectively.

### 2.1. Description of the Model

In this study, the Markov model was used to evaluate the cost-effectiveness of Infliximab, Adalimumab, and Etanercept for treating patients with RA and describing the progression of the disease. As in previous studies, three-month Markov cycles and the time horizon until the end of life were considered.

The Disease Activity Score-28 (DAS-28 due to the evaluation of 28 joints) was used to show the clinical course of the disease. DAS-28 is a standard measure of RA activity, and the score it provides indicates whether the current treatment has worked for the patient. The doctor or nurse calculates the DAS-28 with a special calculator based on several tests, including joint examinations, blood tests, and a self-assessment of how the condition is felt during the investigations. As a rule, the lower the DAS-28 score, the better the patient's condition has been controlled. More severe joint damage is often associated with a higher DAS-28 score [23, 24].  Figure 1 shows a schematic diagram of the Markov model for RA.

The costs and outcomes used in the model were discounted based on the discount rates of 5.8% [25] and 3% [26], respectively. Furthermore, Microsoft Excel and TreeAge Pro softwares were used to analyze the collected data.

### 2.2. Transition Probabilities

All transition probabilities are reported in Table 1, based on the previously published studies.

### 2.3. Cost Data

In this study, the societal perspective was used to extract the costs. The related costs from a societal perspective included direct medical costs (DMC), direct nonmedical costs (DNMC), and indirect costs (IC). DMC related to each of the three medications were retrospectively collected from January 1, 2019, to December 31, 2019, using a researcher-made checklist by referring to the rheumatology department of Hafez Hospital and the personal offices of rheumatologists. DNMC, as well as IC, were also collected using the cost data collection form and the patients' self-report. The human capital approach was applied to calculate the indirect costs.

Furthermore, for international comparisons, the costs were converted into dollars (PPP) using international dollars using a purchasing power parity (PPP) $ exchange rate of 22075 rials per 1 $ rial in 2019 [29].

### 2.4. Utility Data

Utility values were also extracted using the EQ-5D questionnaire, and the health outcomes were evaluated based on quality-adjusted life years (QALY) [30]. To measure the utility scores, we carried out face-to-face interviews or telephone calls with 154 RA patients in 2019.

The interviews were conducted with the outpatients referring to the hospitals and clinics affiliated to Shiraz University of Medical Sciences. It should be noted that an EQ-5D questionnaire is a standard tool for measuring health outcomes, introduced by the EuroQol Group in 1990 (https://euroqol.org/). It includes five questions on five aspects of mobility, self-care, routine activities, pain/discomfort, and anxiety/depression. The respondents' scores range from 0 to 1, and higher scores mean better utility. The patients with RA who were willing to participate in this study were interviewed accordingly. Once the EQ-5D questionnaire was completed, the values of Iran, determined in a separate survey of Goudarzi et al. [31] using time trade-off (TTO), were considered, and the 5-digit codes of the questionnaire were changed to numerical utility.

### 2.5. Incremental Cost-Effectiveness Ratio (ICER)

After obtaining the costs and utilities through the previous steps, the incremental cost-effectiveness ratio (ICER) was calculated using the following formula:

(1) $$\begin{array}{c} \text{ICER}=\frac{\text{Cost}A-\text{Cost}B}{\text{Outcome}A-\text{Outcome}B}. \end{array}$$

### 2.6. Uncertainty Analysis

Finally, the one-way sensitivity analysis and probabilistic sensitivity analysis (PSA) were used to investigate the effects of parameter uncertainty on the results. To do the one-way sensitivity analysis, some critical parameters of the study, such as cost and utility, were changed by 20% for each medication strategy. Then, the results were presented in the form of a Tornado diagram. Also, the PSAs were conducted since the utility and cost variables in the present study were measurable and probabilistic, and they were considered distributions so that beta distribution (*β*) was used to determine the distribution of utility values (0 to 1). The gamma distribution was also used to determine the cost distribution, based on which second-order Monte Carlo simulation was performed using 5000 trials. The PSA results are presented using the cost-effectiveness acceptability curve and the incremental cost-effectiveness scattered plot. The cost-effectiveness acceptability curve is one of the best curves for planning and policy-making. It can help the policymakers and planners of the health system measure the cost-effectiveness probability of each intervention in return for willingness to pay for the expenses. On the other hand, the scatter plot provides more detailed information in individual comparisons. It indicates the percentage of the points in the acceptance area, i.e., below the threshold [32].

An explicit threshold for willingness to pay (WTP) is not available in Iran. Therefore, according to WHO suggestion for developing countries, the willingness to pay was determined as one to three times the gross domestic product (GDP) per capita QALY [33]. GDP was about $ 12547 in Iran in 2019, used as the threshold for willingness to pay [34].

## 3. Results

According to the present study results, a majority of the patients were females (73.37%) and housewives (62.33%), and all the patients had insurance coverage. Besides, 94.34%, 87.5%, and 88.68% of those treated with Infliximab, Adalimumab, and Etanercept were 18-65 years old, respectively. Given that in economic studies, the ages 18 to 65 are considered the productivity ages, they are economically significant.

Table 2 shows the mean costs of RA patients using Infliximab, Adalimumab, and Etanercept. According to this table, the mean direct medical expenses of the patients taking Infliximab, Adalimumab, and Etanercept were $ 9004, $ 10046, and $ 10677, respectively, while the direct nonmedical costs were $ 2484.67, $ 2099.47, and $ 556.76, respectively. Furthermore, the costs of purchasing the primary medication were the highest direct medical costs of the patients using all three medicines (Infliximab: $ 7110.39, Adalimumab: $ 8582.42, and Etanercept: $ 9171.32). The indirect costs were also $ 186.53, $ 192.62, and $ 172.82 (PPP) for the patients taking Infliximab, Adalimumab, and Etanercept.

In general, according to Table 2, the total treatment costs for Infliximab, Adalimumab, and Etanercept were $ 11,675.21, $ 12337.62, and $ 11406.79, respectively. Thus, the cost of treatment with Etanercept was the lowest.

As shown in Table 2, the number of people whose DAS-28 (biologic medication threshold) dropped from 5.1 to <2.6 was 27 (51%), 33 (68.75%), and 29 (54.72%) in the case of Infliximab, Adalimumab, and Etanercept, respectively.

According to QALY, the highest utility scores of the patients with RA obtained from the EQ5D questionnaire were those of the patients using Etanercept who had DAS-28 < 2.6 (0.891).

As shown in Figure 2 and Table 3, the results of utility cost analysis using the Markov model showed that the mean costs and QALY in Infliximab, Adalimumab, and Etanercept arms were $ 79,518.33 and 12.34, $ 91,695.59 and 13.25, and $ 87,440.92 and 11.79, respectively. These results indicate that treatment with Infliximab or Adalimumab was predominant over treatment with Etanercept and was more cost-effective. However, the cost-effectiveness ratio calculated for Adalimumab treatment compared to Infliximab was $ 13,420.09, suggesting that $ 13,420.09 had to be spent for each additional QALY in the patients treated with Adalimumab. In this case, ICER had to be compared with the threshold to decide. The method provided by the WHO was used to calculate the threshold; thus, if the ICER were lower than one times GDP per capita, the program would be much cost-effective, and if it were lower than three times GDP per capita, the program would be cost-effective [33]. The GDP per capita was $ 12547 in 2019 [34]. Besides, considering that the ICER was $ 13,420.09, more than one times GDP per capita, Adalimumab treatment was not more cost-effective than Infliximab treatment due to the ICER of over one times threshold.

### 3.1. Uncertainty Analysis

#### 3.1.1. One-Way Sensitivity Analysis

Figure 3 shows the percentage of change in the incremental cost-effectiveness ratio in treating Infliximab vs. Adalimumab. The total cost-effectiveness ratio is also presented with $ 13,420.12. According to the Tornado diagram results, ICER had the highest sensitivity to the reduction of utility in the treatment with Adalimumab in remission mode and the minor sensitivity to the decrease in other costs of Adalimumab in the weak state of the disease. Therefore, if utility in the treatment with Adalimumab changes in remission mode, considering that the ICER value will still become a positive number, it cannot be decided with certainty that Infliximab has superiority over Adalimumab.

Figure 4 shows the percentage of change in the incremental cost-effectiveness ratio of Infliximab treatment compared to the treatment with Etanercept. The number $ -14,348.30 indicates the incremental cost-effectiveness ratio. The Tornado diagram results show that ICER was the most sensitive to reducing utility in treatment with Infliximab in an intermediate state and had the least sensitivity to the reduction of other utilities of the Infliximab in the low and remission states. Furthermore, given that in this case, the ICER value was again negative, it could be decided with certainty that Infliximab was superior to Etanercept.

### 3.2. Probabilistic Sensitivity Analysis (PSA)

The PSA results were uncertainly presented using the cost-effectiveness acceptability curve and the incremental cost-effectiveness scattered plot. The acceptability curve result based on QALY shows that Infliximab was below the cost-effectiveness threshold of $ 12547 PPP (one times GDP) in 77% of the simulations and, therefore, was the most cost-effective medication therapy strategy (Figure 5).

In addition, the results of the scatter plots based on QALY (Figures 6(a) and 6(b)) showed that compared to Adalimumab and Etanercept, Infliximab was in the acceptance area and below the threshold in 81% and 91% of the simulations, respectively. This result indicates lower cost- and higher effectiveness than the other two alternatives and, therefore, is a more cost-effective strategy.

## 4. Discussion

For the first time, this study was conducted to evaluate the cost-effectiveness of Infliximab, Adalimumab, and Etanercept in patients with RA in Iran. This study is aimed at comparing three medicines that act against TNF-alpha, which was widely used to treat RA. All three medicines are considered equally effective in terms of clinical value for physicians, and the main difference is in their price. Therefore, the subject of the present study was which ones are more cost-effective used against TNF-alpha? All three medicines studied in this research are used subcutaneously through an autoinjector pen and are no different in this regard.

According to the present study findings, treatment with Infliximab, Adalimumab, and Etanercept had a mean cost of $ 11,675.21, $ 12,337.62, and $ 11,406.79 PPP, respectively, for each one-year treatment course. Thus, the mean treatment cost per patient taking Etanercept was lower than treatment with the two other medications. In this regard, the results are consistent with those of the studies by Tang et al., Carter et al., and Ramírez-Herráiz et al. [35–37].

The DMC, DNMC, and IC of the patients using Infliximab were $ 9004.00 (77.12% of the total costs), $ 2484.67 (21.28% of the total costs), and $ 186.53 (1.60% of the total costs) PPP, respectively. However, the prices of patients paid for Adalimumab were $ 10045.53 (81.42% of the total costs), $ 2099.47 (17.02% of the total costs), and $ 192.62 (1.56% of the total costs) PPP, respectively, and those of the patients paid for taking Etanercept were $ 10677.20 (93.60% of the total costs), $ 556.76 (4.88% of the total costs), and $ 172.82 (1.52% of the total costs) PPP. Meanwhile, the cost of purchasing the primary medication was the highest direct medical cost of the patients using all the three medications (Infliximab: $ 7110.39 PPP (78.97% of the total costs); Adalimumab: $ 8582.42 PPP (85.44% of the total costs); and Etanercept: $ 9171.32 PPP (85.90% of the total costs)). The results of this study are consistent with those of Incerti et al., Soini et al., Bonafede et al., Lekander et al., and Saraux et al. [38–42].

The results of this study showed that the number of the patients whose DAS-28 dropped from 5.1 (biologic medication threshold) to <2.6 in the Infliximab, Adalimumab, and Etanercept groups was 27 (51%), 33 (68.75%), and 29 (54.72%), respectively. This result indicates that Adalimumab was the most effective medication.

A study carried out by Cárdenas et al. examined the cost-effectiveness of Infliximab, Adalimumab, and Etanercept over two years showing that Adalimumab was more effective than the other two medications [43]. Furthermore, the results of the study by Wiens et al. that entitled the analysis of effectiveness and safety of Adalimumab, Etanercept, and Infliximab for the treatment of RA indicated that short-term therapy with Etanercept and Adalimumab was most effective, while long-term treatment with Adalimumab was the most effective [44].

In a study entitled direct comparison of therapeutic responses, disease control, and medication adherence in patients with RA treated with Adalimumab, Etanercept, and Infliximab, Hetland et al. (2009) concluded that Infliximab had the lowest therapeutic response, the lowest rate of recovery, and the lowest rate of medication adherence. However, Adalimumab had the highest therapeutic response and remission rate, while Etanercept had the highest medication adherence [45]. In this respect, the results are consistent with the findings of the present study.

The study results by Santos-Moreno et al. conducted as a cohort in Colombia to directly compare the effectiveness of Adalimumab, Etanercept, and Infliximab showed that in the beginning, the DAS-28 was 4.1 but it changed to 2.39 after 36 months. The most common complication was dermatitis. It was finally concluded that all three medications reduced the severity of the disease, and Etanercept had a lower incidence of side effects than the other two medications. It is in line with the present study regarding the effectiveness of all three medications in reducing the symptoms and controlling the disease [46].

According to the present study results, the highest utility of each medication was found in the patients with DAS-28 < 2.6, and as the Disease Activity Score-28 (DAS-28) increased, the life desirability decreased. As the Disease Activity Score-28 (DAS-28) increased, more joints got involved in the disease, and the effect of the medications was usually reduced. Therefore, the patients entered the severe phase of the disease, and it could be natural that their life desirability decreased [47].

The cost-utility analysis results using the Markov model showed that the mean costs and QALY amount in the Infliximab, Adalimumab, and Etanercept arms were $ 79,518.33 and 12.34, $ 91,695.59 and 13.25, and $ 87,440.92 and 11.79, respectively. Thus, treatment with Infliximab or Adalimumab was predominant over Etanercept and was also more effective. Besides, the comparison of the threshold introduced by the WHO (one times GDP-per capita) and the incremental cost-effectiveness ratio (ICER) was obtained by comparing Adalimumab and Infliximab indicated that Infliximab was a more cost-effective option.

In their study entitled cost analysis and application of second-line treatment with Rituximab in comparison with Tumor Necrosis Factor Inhibitors in RA, Lopatina et al. showed that over a one-year time horizon, Rituximab and Etanercept resulted in the effectiveness of 0.80 QALYs with the costs of $ 14,291 and $ 18,880, respectively. They were the dominant choices compared to Adalimumab ($ 0.79 QALYs, $ 18,825) and Infliximab (0.76 QALYs, $ 20158). Also, over a 6-year time horizon, Rituximab (4.42 QALYs ($ 82,402) was predominant compared to Adalimumab (4.30 QALYs, $ 101,420), Etanercept (4.02 QALYs, $ 99,191), and Infliximab (3.71 QALYs, $ 100,396). In a probabilistic analysis, Rituximab was predominant over Adalimumab, Etanercept, and Infliximab with the probabilities of 0.51, 0.62, and 0.65, respectively [48].

Zrubka et al. conducted a systematic study and evaluated the long-term efficacy and cost-effectiveness of Infliximab as a first-line treatment for RA. The results showed that the recovery of the RA patients treated with Infliximab was significant within six months compared to the control group. Over a year, the improvement was remarkable in those who used Infliximab than the control strategies [47]. In this respect, the results are consistent with those of the present study.

In Taiwan, Chen et al. examined the cost-effectiveness of Tofacitinib vs. Adalimumab and concluded that the QALY obtained in treatment with Tofacitinib was 0.09 more than Adalimumab (5.13 vs. 5.04). Besides, the incremental cost-effectiveness was 143122 QALY/$ NT. The one-way sensitivity analysis confirmed that the results were robust [49]. These results are in line with those of the present study.

Fatemi et al. conducted a study in Iran and examined the cost-effectiveness of Tofacitinib vs. Adalimumab and Etanercept. They concluded that Tofacitinib was more cost-effective than the two others, and although Tofacitinib had fewer QALYs than Etanercept (6.664 vs. 6.876), it cost less on the lifetime horizon ($ 42,565.04 vs. $ 58,696.29). Tofacitinib also cost less than Adalimumab ($ 50,299.91 vs. $ 51,550.29) and had more QALYs (6,900 vs. 6,687). The sensitivity analysis also showed that the results were sensitive to the cost of the medications [50]. These findings are in line with those of the present study.

In a study in Brazil entitled the cost-effectiveness analysis of RA medications, dos-Santos et al. suggested that Golimumab was the most effective medication. It was also the dominant option compared to Etanercept. On the other hand, the Adalimumab ICUR was $ 95,095.37. The sensitivity analysis indicated that the results were robust [51].

The results of a study by Chastek et al. on the comparative efficacy of TNF blockers in RA patients treated with Adalimumab, Etanercept, and Infliximab from January 1, 2006, to 2008 showed that Etanercept had the lowest dose and the patients showed the best response to Infliximab [52]. This study is in line with the results of the present study.

In their study entitled “biological medications for RA in Medicare: Cost-Effectiveness Analysis”, Wailoo et al. concluded that the efficacy of Infliximab, Adalimumab, and Etanercept in the treatment population was similar, but Infliximab was more costly [53]. This conclusion might be due to the higher price of this medication.

Curtis et al. conducted a study on the cost-effectiveness of biological medications in RA patients with commercial insurance, in which the subjects were 18 to 63 years old. They finally indicated that Etanercept was the most cost-effective option [54]. Their study results are inconsistent with the present research, which could be the lower price of Etanercept compared to other medications.

Also, the one-way sensitivity analysis results on Infliximab and Etanercept confirmed the robustness of the study results and indicated that Infliximab could be a superior medication compared to Etanercept.

The probabilistic sensitivity analysis results showed that on the cost-effectiveness acceptability curve, Infliximab was in the acceptance area and below the threshold in 77% of the simulations. The medication was also in the acceptance area of cost-effectiveness scattered plot, e.g., below the threshold in 81% and 91% of the simulations compared to Adalimumab and Etanercept. This finding indicates its lower costs and higher effectiveness than the other two alternatives, and therefore, the strategy was more cost-effective.

The present study had some limitations as the limited data required, especially for the disease transition probabilities. Hence, fixed rates were used in this study. In addition, intangible costs were not calculated in this study due to the impossibility of measuring them accurately.

Regarding the generalizability of the results, it can be said that since the medications are used in all provinces and medical centers of Iran to treat RA patients and their prices are the same throughout the country, the results of this study can be generalized to other provinces and the whole country. However, it is necessary to consider the following items to generalize the results to other countries: epidemiology of the disease and demographic structure, existence of resources, prices, evaluation of outcomes by individuals, threshold, and the use of various effectiveness indicators in different studies that may affect the results of the present study. Therefore, caution is needed when generalizing the results to other countries.

According to the results of this study, Infliximab was more cost-effective than the other two medications. Therefore, based on the sensitivity analysis results, as long as the study parameters do not change significantly, it is suggested that Infliximab should be used as the priority for treating patients with RA. Also, health policymakers and managers should try to increase insurance coverage and reduce out-of-pocket payments.

## Figures and Tables

**Figure 1:** Schematic design of the Markov model for rheumatoid arthritis. Rem: remission; Lo: low; Mod: moderate; Sev: severe.

**Figure 2:** Cost-effectiveness plan for treatment with Infliximab, Adalimumab, and Etanercept in patients with RA.

**Figure 3:** Tornado diagram for one-way sensitivity analysis of Infliximab and Adalimumab treatments. ifx: Infliximab; ada: Adalimumab; rem: Remission; mod: moderate; sev: severe; eff: effectiveness; c: cost.

**Figure 4:** Tornado diagram of one-way sensitivity analysis for Infliximab and Etanercept treatments. ifx: Infliximab; eta: Etanercept; rem: Remission; mod: moderate; sev: severe; eff: effectiveness; c: cost.

**Figure 5:** Cost-effectiveness acceptability curve of Infliximab, Adalimumab, and Etanercept obtained through Monte Carlo simulation.

**Figure 6:** Scatter plot of incremental cost-effectiveness of Infliximab compared with Adalimumab and Etanercept.

**Table 1:** Transition probabilities used in the Markov decision model.

Stage	Remission	Low	Moderate	Severe	Death
Remission	0.500	0.310	0.119	0.070	0.001
Low	0.262	0.388	0.306	0.040	0.004
Moderate	0.070	0.217	0.550	0.155	0.008
Severe	0.020	0.040	0.307	0.621	0.012
Source	[27]				[28]

**Table 2:** Mean costs and utility of rheumatoid arthritis patients using Infliximab, Adalimumab, and Etanercept (in terms of purchasing power parity).

Costs	Infliximab		Adalimumab		Etanercept	
	PPP	%	PPP	%	PPP	%
Direct medical cost						
Visits	172.14	1.91	172.14	1.71	172.14	1.61
Medication	7110.39	78.97	8582.42	85.44	9171.32	85.90
Tests	618.40	6.87	618.40	6.16	618.40	5.79
Physiotherapy and other expenses	410.41	4.56	387.60	3.86	439.37	4.03
Diagnostic services	284.96	3.16	284.96	2.84	284.96	2.67
Injection cost	407.70	4.53	0.00	0.00	0.00	0.00
Total	9004.00	77.12	10045.53	81.42	10677.20	93.60
Direct nonmedical cost						
Transportation	1451.79	58.43	1285.51	61.23	318.02	57.12
Accommodation	580.92	23.38	435.22	20.73	125.22	22.49
Meals	451.96	18.19	378.74	18.04	113.52	20.39
Total	2484.67	21.28	2099.47	17.02	556.76	4.88
Indirect cost						
Lost revenue	186.53	1.60	192.62	1.56	172.82	1.52
Total cost	11675.21	100	12337.62	100	11406.79	100
Effectiveness	Number	%	Number	%	Number	%
DAS‐28 < 2.6	27	50.94	33	68.75	29	54.72
2.6 < DAS‐28 < 3.2	17	32.07	2	4.2	5	9.43
DAS-28 > 3.2	9	16.98	13	27.08	19	38.85
Utilities	Mean	Sd	Mean	Sd	Mean	Sd
DAS-28 < 2.6	0.836	0.196	0.725	0.193	0.891	0.126
2.6 < DAS‐28 < 3.2	0.717	0.148	0.656	0.223	0.337	0.276
3.2 < DAS‐28 < 5.1	0.23	0.216	0.437	0.209	0.391	0.211
DAS-28 > 5.1	0.2	0.170	0.23	0.190	0.223	0.190

**Table 3:** Results of cost-utility analysis for rheumatoid arthritis patients treated with Infliximab, Adalimumab, and Etanercept.

Strategy name	Cost (PPP$)	QALYs	Incremental cost	Incremental utility	ICER (incremental cost per QALY gained) PPP$
Infliximab	79,518.33	12.34	0.00	0.00	0.00
Etanercept	87,440.92	11.79	7,922.59	-0.55214	Abs. Dominated
Adalimumab	91,695.59	13.25	12,177.26	0.90739	13420.09

## Data Availability

All data used to support the findings of this study are included within the article.
